# Effects of a pre-visit educational website on information recall and needs fulfilment in breast cancer genetic counselling, a randomized controlled trial

This article has been retracted.

**DOI:** 10.1186/bcr3133

**Published:** 2012-03-06

**Authors:** Akke Albada, Sandra van Dulmen, Jozien M Bensing, Margreet GEM Ausems

**Affiliations:** 1 NIVEL (Netherlands Institute for Health Services Research), Otterstraat 118-124, Utrecht, 3500 BN, the Netherlands; 2 Department of Primary and Community Care, Radboud University Nijmegen Medical Centre, Geert Grooteplein-Noord 21, Nijmegen, 6525 EZ, the Netherlands; 3 Department of Psychology, Utrecht University, Heidelberglaan 1, Utrecht, 3584 CS, the Netherlands; 4 Department of Medical Genetics, University Medical Center Utrecht, Lundlaan 6, 3508 AB, the Netherlands

## Abstract

**Introduction:**

Pre-visit education which helps counselees to prepare for their first visit for breast cancer genetic counseling might enhance information recall and needs fulfilment. This study assessed the effects of a pre-visit website with tailored information and question prompt sheet (QPS), named E-info gene^ca^.

**Methods:**

A total of 197 counselees were randomized to receive usual care (UC) or UC plus E-info gene^ca^. All counselees completed a pre- and post-visit questionnaire and visits were videotaped. We studied effects on counselees' information recall, knowledge about breast cancer and heredity, fulfillment of needs, risk perception alignment, anxiety and perceived personal control, using multilevel regression analyses.

**Results:**

Intent-to-treat analysis showed that counselees in the intervention group (*n *= 103) had higher levels of recall of information from the consultation (β = .32; confidence interval (CI): .04 to .60; *P *= .02; d = .17) and post-visit knowledge of breast cancer and heredity (β = .30; CI: .03 to .57; *P *= .03) than counselees in the UC group (*n *= 94). Also, intervention group counselees reported better fulfilment of information needs (β = .31; CI: .03 to .60; *P *= .03). The effects of the intervention were strongest for those counselees who did not receive an indication for DNA testing. Their recall scores showed a larger increase (β = .95; CI: .32 to 1.59; *P *= .003; d = .30) and their anxiety levels dropped more in the intervention compared to the UC group (β = -.60; CI: -1.12 to -.09; *P *= .02). No intervention effects were found after the first visit on risk perception alignment or perceived personal control.

**Conclusions:**

This study shows that pre-counseling education, using tailored information technology, leads to more effective first visits for breast cancer genetic counseling, in particular for counselees who received no indication for DNA testing and, therefore, had no indication for a second visit. Future study should focus on the effects of a pre-visit website on the outcomes after a complete series of visits.

**Trial registration:**

Dutch Trial Register ISRCTN82643064.

## Introduction

Women who are diagnosed with breast cancer or have affected relatives often worry about their or their children's risk to (re)develop breast cancer. Therefore, they might be referred to genetic counseling. Breast cancer genetic counseling aims to educate individuals about their breast cancer risk to optimize risk management, increase personal control and decrease anxiety [1]. However, studies have consistently found that most counselees still have a marked overestimation of risks relative to counselors' evaluations after genetic counseling [2]. The aims of the first visit are mainly to educate the counselee about breast cancer and genetics, make a risk estimation and decide whether a DNA test is indicated. For counselees who are the first in their family to request breast cancer genetic counseling, an indication for a DNA test might be for themselves or an affected relative. These counselees are assigned with the transmission of information regarding this possible indication, breast cancer risks and preventive options to their relatives. Counselees are unlikely to transfer and act according to advice that they do not remember [3]. Their recall of information from the first visit is, therefore, especially important for the course of breast cancer genetic counseling and the risk management of themselves and their relatives. However, after the initial visit counselees show only small improvements in knowledge about breast cancer and genetics [4,5], risk perceptions, perceived personal control and anxiety [5] and their recall of information has not been studied yet.

Generally, recall of information from medical visits is low. Kessels [6] reported that 40% to 80% of the information presented was forgotten immediately by patients. Studies in oncology found that patients recalled only half of the information provided in general oncology visits when they were cued with topics [7] and actively reproduced only 23% of the information from consultations about chemotherapy [3]. Cued recall within genetic counseling for diverse disorders was higher, namely three-quarters of the most important items [8]. These higher scores might be due to the percentages of patients who request genetic counseling at their own initiative because of a need for information. Alternatively, different ways to assess recall might result in higher estimates [3].

Unidirectional transfer of generic instead of tailored or counselee-specific information has long been the preferred method in cancer genetics, both in the consultation and in pre-visit information. However, counselee-specific information is expected to be more effective in reaching the aims of counseling by increasing the counselee's recall [9,10]. Tailoring information to individual needs is an effective way of reducing the amount of information and ensuring that only relevant information is provided [11]. According to the Elaboration Likelihood Model and confirmed by findings from neuropsychological research, increased personal relevance of information enhances central processing [12] and information retrieval [13,14]. Therefore, the use of counselee-specific rather than general recommendations should enhance recall [15]. Additionally, the provision of additional written information and spreading information over different time points might show increased retention [14,16,17]. The combination of pre-visit tailored information with more counselee-specific information provided during the visit, might thus result in increased information recall and knowledge. Additionally, improved recall of the risk information might increase the alignment of counselees' risk perception with the counselors' estimation.

Previous studies of computer-based education prior to genetic counseling were limited to assessment of counselees' knowledge about breast cancer and heredity [18-20]. The current study assessed counselee's recall of the counselor's advice as discussed during the visit. Comparison with the consultation video determined whether this recall was correct. As opposed to general knowledge of hereditary breast cancer this recall of the counselor's explanation and advice determines whether counselees can transfer risk estimates correctly to relatives and can act upon the advice given [7]. Additionally, fulfillment of information needs evaluates whether the counselee's agenda was met. Studies that evaluated the impact of meeting counselees' individual needs found that [21] adjusting communication to these needs resulted in improved counselee's perceived personal control and anxiety [5].

This article describes an randomized controlled trial (RCT) focused on the effects of a pre-visit educational website, E-info gene^ca ^[22] to optimize the first visit. The website provided computer-tailored information concerning counselees' pre-visit needs, for example, the procedure and consequences of genetic counseling for counselees who were the first in their family to request breast cancer genetic counseling [23]. Additionally, the website offered a QPS to encourage counselees to formulate questions [24]. These questions were sent ahead to the counselor and were answered during the visit. Previous studies showed that after having accessed E-info gene^ca^, counselees communicated more assertively by more often sharing their agenda, directing the flow of the visit and paraphrasing the counselor to check their understanding. As a result, counselors provided more counselee-specific information [25]. The current study evaluates whether the pre-visit educational website improved counselee outcomes after their first visit, that is, information recall, knowledge, fulfillment of needs, risk perception alignment, anxiety and perceived personal control.

## Methods

### Study design

This study was conducted at the department of Medical Genetics of the University Medical Center (UMC) Utrecht. The study was approved by the institutional medical ethical committee and is registered in the Dutch Trial Register (ISRCTN82643064). The department of Medical Genetics enrolled counselees from February 2008 to April 2010. This department offers breast cancer genetic counseling according to the Dutch guidelines [26] and services are similar to those of the other eight family cancer clinics in the Netherlands. New counselees, 18 years old or older, who were the first in their family to seek breast cancer genetic counseling, were sent information about the study and an opt-out form. The opt-out form included a question about reasons for withdrawal. Counselees were ineligible if they lacked internet or email access or when they requested pre-symptomatic DNA testing in the presence of an identified *BRCA1/2 *gene mutation in a relative. All counselees who did not return the opt-out form were randomly assigned 1:1 to the usual care (UC) or intervention group (UC + website E-info gene^ca^) by a secretary unaware of respondent's characteristics using sequentially numbered, sealed, opaque envelopes. UC comprised a brief standard pre-visit leaflet with information about the counseling procedure. Both UC and intervention group respondents received a login to access the web-based baseline questionnaire. Upon completion of the baseline questionnaire the intervention group respondents received a link to access the website E-info gene^ca^. At the start of the consultation the counselor collected the informed consent form. The visits were videotaped. In the week after their visit, counselees again completed a web-based questionnaire. Because with 100 counselees in each group, there was an 80% power to detect effect sizes of d = .40 or higher, we aimed to include 200 counselees.

### Counselor characteristics

Counselors were clinical geneticists, residents in clinical genetics, genetic counselors or genetic counselors in training. All will be referred to as 'counselor'. Their age, gender and number of years of experience with cancer genetic counseling was assessed at the start of their participation in the study.

### Counselee characteristics

Age, having children, personal and family cancer history and educational attainments were assessed in the baseline counselee questionnaire. All but the latter were derived from the medical file if missing. Additionally, whether or not there was an indication for DNA testing for the counselee or an affected family member was collected from the medical files.

### Measures

Counselees' recall of information from the visit was assessed in the post-visit questionnaire with seven questions for cued recall. Each question prompted a topic of the consultation, for example, limitations of DNA testing and involving family members, and these topics were based on the counselees' information needs questionnaire Quote-gene^ca ^[23]. Each question started with a multiple choice indication of whether the topic was discussed. Answer options were 1) no, not discussed, 2) yes it was discussed but I don't remember what was said, 3) yes, namely. With the latter, the counselee was invited to write down what she recalled about this topic [3].

Coders first assessed whether the topic was discussed in the visit based on the videotapes. Second, each item recalled was compared with the specific items mentioned by the counselor [3,7]. The percentage of accurate recall was calculated by dividing the sum of the accurately recalled items by the total number of items discussed [7].

Recall was coded by AA and a second coder recoded a random 10% of the visits. Coders were blinded to group allocation. Interrater reliability was assessed. Cohen's kappa for the recall per item averaged 0.70 (range 0.39 to 1.0). The intra class correlation (ICC) of the overall recall percentage was 0.89.

The level of accurate knowledge about hereditary breast cancer was assessed using the validated Dutch hereditary breast cancer knowledge scale [5,27]. Respondents indicated whether each item was correct, incorrect, or whether they did not know. A knowledge score was computed as the mean number of correct answers, with higher scores indicating more accurate knowledge.

Pre-visit, counselees' needs were assessed with the QUality Of counselling Through counselees' Eyes scale for cancer genetic counseling (QUOTE-gene^ca^) [23]. At baseline, respondents indicated the importance (not important, fairly important, important, extremely important) of these needs. Post-visit, identical items were administered to measure fulfillment of these needs (inadequate, not really adequate, adequate, more than adequate) [28]. The QUOTE-gene^ca ^includes four generic needs, which refer to what a counselor should do during counseling (25 items) and four cancer genetic information needs, which refer to receiving explanations on hereditary cancer (19 items), as identified by principal component analysis with good internal consistency [23].

Risk perception alignment was defined as the degree of agreement of the counselee's risk perception with the counseled risk [2]. Counselees rated their perceived risk that they themselves would (re-) develop breast cancer in the future, that hereditary breast cancer runs in their family and that they themselves had inherited a breast cancer gene mutation, on visual analogue scales from 0 to 100%. Counselors rated their estimations of these risks for the counselee on identical scales after the visit. Additionally, we categorized this risk based on population or slightly increased (< 20%), moderate (17% to 30%) or high risk (> 30%) of developing breast cancer [29]. The perceived absolute risk of developing breast cancer was assessed on a 5-point scale from 1 'very low to 5 'very high'. Finally, the perceived relative risk was assessed, indicating whether the counselee perceives her breast cancer risk as lower, even or higher than the average risk for women of her age [30].

Pre- and post-visit anxiety was assessed with the validated Dutch state version of State-Trait Anxiety Inventory (STAI; 10 items) [28,31]. Scores range from 10 to 40, higher scores indicating greater anxiety.

Pre- and post-visit perceived control was assessed using the validated Dutch version of the Perceived Personal Control questionnaire (PPC) [28,32]. Scores range from 0 to 2 with high scores indicating high perceived control.

### Analysis

We analyzed respondents in the groups to which they were randomized regardless of whether they actually accessed E-info gene^ca ^or other protocol irregularities. The few missing values (seven cases) on the baseline measures of educational attainment were imputed with the median. Post-visit, the number of missing data on the outcome variables ranged from 18 for knowledge and recall, 20 for fulfillment, 22 for perceived personal control, 25 for anxiety and 43 for risk perception. All counselees were included in analyses through use of repeated measures analysis which makes use of available data of all cases (intention-to-treat analysis) [33].

Intervention and UC group counselees were compared on socio-demographics, cancer history and levels of pre-visit measures using Chi-square tests and t-tests. To account for the multilevel structure of measurements (level 1) nested within counselees (level 2) nested within counselors (level 3), random effects multilevel regression analyses were conducted. This method corrects for the number of consultations per counselor [34]. The percentage of variance explained at the counselor level ranged from zero for knowledge to 12% for anxiety. Analyses were controlled for baseline values, counselee disease status, education and receiving an indication for DNA testing. Additionally, analyses were controlled for background variables at the counselor level, namely whether the counselor was a clinical geneticist or a genetic counselor and whether or not the counselor was still in training. All analyses were conducted using Stata 10. Two-sided tests of significance were performed and results were considered statistically significant when *P *< .05. Furthermore, Cohen's effect sizes (d) were calculated [35].

## Results

### Response

Few counselees were ineligible because of lack of internet or email access (24 of 371; 6.5%). The response was 58.6%. Half of the decliners gave a reason (72 of 139; 50.4%). Most decliners preferred that the visit not be videotaped (48 of 72; 66.7%). There were no significant differences between participants and decliners in age (t = 1.62; *P *= .11), disease status (*X^2 ^*= .05; *P *= .81), family history of cancer (*X^2 ^*= .06; *P *= .82) and referral pathway (*X^2 ^*= 87; *P *= .35). A flowchart of the study and reasons for non-response are shown in Figure 1.

**Figure 1:** **Flow diagram of study participants**.

### Counselors

All fourteen breast cancer genetic counselors of the department of Medical Genetics participated and recorded 4 to 29 consultations each. Six were genetic counselors, of whom three were in training (all women). Three were experienced (5 to 15 years) clinical geneticists (two men, one woman) and five were clinical geneticists in training (all women), see Table 1.

**Table 1:** Characteristics of the genetic counsellors (*N *= 14).

	Mean	SD (range)
Age (years)	36.22	9.60 (26 - 53)
	
	**N**	
	
Genetic counselor	3	
Genetic counselor in training	3	
Clinical geneticists	3	
Clinical geneticist in training (resident)	5	
		
Male	2	
Female	12	
		
Experience in cancer genetic counseling		
< 1 year	8	
1 to 5 years	1	
> 5 years	3	
5 to 10 years	0	
> 10 years	2	

### Counselee characteristics

As shown in Table 2 UC and intervention group respondents were similar with regard to all background characteristics except for being affected with breast cancer themselves (*X^2 ^*= 5.10; *P *= .02). There was no significant association between having (had) breast cancer and baseline knowledge (T = .12; *P *= .91). One counselee was affected with ovarian cancer. There were no significant baseline differences in knowledge, information needs, risk perception, anxiety and perceived personal control between the study groups (Tables 3, 4 and 5).

**Table 2:** Counselee characteristics (*N *= 197).

	UC group (*n *= 94)		Intervention group (*n *= 103)	
	**Mean**	**SD (range)**	**Mean**	**SD (range)**

Age (years)	41.3	11.5 (21 to 68)	41.5	11.3 (21 to 69)
	N	%	N	%
	
Children (having children)	64	68.1	71	68.9
Personal history of breast cancer (affected)	29	30.9	49	47.5
1^st ^degree relatives affected with breast cancer	47	52.8	54	52.9
Educational attainment:				
University (MSc/BSc)/higher vocational education (BSc)	42	48.8	35	35.34
Middle vocational education	23	26.7	30	30.3
High school/Secondary education	18	20.9	33	33.3
< High school level	3	3.5	1	1.0
Referral pathway:				
GP	50	55.6	44	43.1
Specialist consultant UMC	18	24.4	32	31.4
Specialist consultant peripheral hospital	21	20.0	26	25.5
				
Indication for DNA-testing^a^	67	71.3	81	78.6
Breast cancer risk category:				
High (≥ 30% lifetime risk)	17	18.1	18	17.5
Moderate (20 to 30% lifetime risk)	34	36.2	38	36.9
Population (< 20% lifetime risk)	43	45.8	47	45.6

^a ^Indication for testing the counselee or a relative as judged during the initial visit. Summations vary due to missing values. GP, general practitioner; UC, usual care; UMC, University Medical Center.

**Table 3:** Counselees' level of accurate knowledge about breast cancer and heredity.

	Baseline (T0)				Post-visit (T1)				
	
	UC group (*n *= 94)		Intervention group (*n *= 103)		UC group (*n *= 94)		Intervention group (*n *= 103)		
***Scale***	**Mean**	**SD**	**Mean**	**SD**	**Mean**	**SD**	**Mean**	**SD**	***P* ^a^**

Accurate knowledge score (0-7)	4.65	1.46	4.64	1.60	5.71	1.53	6.10	1.13	**.03**
	
True/false knowledge items:	correct answer		correct answer		correct answer		correct answer		
	
	n	%	n	%	n	%	n	%	
	
Early detection and treatment of bc lead to longer survival than late detection and treatment (True)	86	96.6	98	97.0	79	94.1	90	94.7	.74
All women who are carrier of an altered gene (mutation) for bc, will develop bc in the long term (False)	39	43.8	47	46.5	56	66.7	72	75.8	**.048**
A woman who has a sister with an altered gene (mutation) for bc, has a 50% change (1 in 2) to also carry the mutation herself (True)	31	35.2	34	33.7	52	61.9	70	73.7	.09
A woman who does not have an altered gene (mutation) for bc, can nevertheless develop bc (True)	70	78.7	77	77.8	78	92.9	89	93.7	.74
Physical examination is necessary only when you have complaints; at that point it is soon enough to prevent bc (False)	84	94.4	93	93.0	76	90.1	89	93.7	.56
If a father has an altered gene (mutation) for bc, then his children have 50% chance (1 in 2) of also having this mutation (True)	27	30.3	38	37.6	60	71.4	81	85.3	**.02**
If in a family, in which bc frequently occurs, no altered gene (mutation) for bc is found, then regular breast surveillance is no longer necessary (False)	77	86.5	82	81.2	79	94.1	88	92.6	.50

^a ^Between group differences at T1. bc, breast cancer; UC, usual care.

**Table 4:** Counselees' information needs at baseline and fulfilment of these needs concerning breast cancer genetic counselling post-visit.

	Baseline (T0) needs				Post-visit (T1) fulfilment				
		
	UC group (*n *= 94)		Intervention group (*n *= 103)		UC group (*n *= 94)		Intervention group (*n *= 103)		
		
Scale (1-4) Factors (1-4)	Mean	SD	Mean	SD	Mean	SD	Mean	SD	*P* ^a^
Cancer genetic information needs	3.24	.38	3.25	.39	3.02	.55	3.14	.53	**.03**
Determination and meaning of being a carrier of a cancer gene	3.32	.47	3.33	.49	3.03	.62	3.15	.58	**.04**
Emotional consequences for counselee and family	3.13	.55	3.08	.59	2.88	.69	2.97	.67	.26
Own risk of developing breast cancer	3.44	.47	3.46	.56	2.92	.74	2.99	.77	.36
Heredity of breast cancer	2.67	.53	2.80	.53	3.25	.59	3.44	.53	**.008**
Generic needs	3.25	.36	3.25	.37	3.21	.44	3.26	.43	.22
Procedural aspects of counseling	2.93	.52	2.82	.58	3.08	.46	3.14	.52	.23
Sensitive communication	2.72	.74	2.65	.79	3.46	.47	3.50	.43	.53
Emotional support	2.93	.53	2.90	.62	3.04	.55	3.06	.49	.46
Assessment of susceptibility	3.09	.54	3.1	.49	3.03	.62	3.12	.59	.17

^a ^Between group differences at T1. UC, usual care.

**Table 5:** Effects of E-info gene^ca ^on risk perception, anxiety and perceived personal control.

		Baseline (T0)		Post-visit (T1)				
		**UC group** **(*n *= 94)**	**Intervention group (*n *= 103)**	**UC group** **(*n *= 94)**	**Intervention group (*n *= 103)**			
	**Range**	**Mean (SD)**	**Mean** **(SD)**	**Mean (SD)**	**Mean** **(SD)**	**B^a^**	***P* ^a^**	**d^a^**

Anxiety (10-40)	10.0 - 40.0	19.94 (6.25)	19.73 (5.81)	18.54 (6.11)	17.91 (5.58)	-.70	.24	.11
Perceived personal control (1-3)	.22 -2.00	1.23 (.43)	1.15 (.41)	1.33 (.41)	1.34 (.44)	-.03	.49	.00
Breast cancer risk perception alignment (mean difference between counselee and counselor's risk estimation)	1-100	26.69 (19.89)	27.83 (18.20)	18.00 (16.17)	16.81 (16.35)	.07	.79	.07
No indication for DNA-testing (*n *= 49): Anxiety	10-34	20.52 (6.76)	20.00 (6.50)	19.15 (7.96)	16.65 (5.49)	**-.60**	**.02**	**.36**
Perceived personal control (1-3)	.22 -2.00	1.37 (.41)	1.19 (.46)	1.25 (.49)	1.19 (.59)	.09	.83	.00
Breast cancer risk perception alignment (mean difference between counselee and counselor's risk estimation)	1-100	29.75 (20.87)	25.94 (15.69)	12.37 (20.27)	11.32 (17.59)	-.08	.79	.06

^a ^Between group difference at T1. UC, usual care.

### Information recall

Less than half of all information items were recalled correctly (Table 6). The total number of recalled items was significantly higher in the intervention compared to the UC group (β = .32; CI: .04 to .60; *P *= .02; d = .17). The effect size of the intervention was larger for the counselees who did not receive an indication for DNA testing (β = .95; CI: .32 to 1.59; *P *= .003; 52.69(23.72) versus 59.94(25.09); d = .30). The educational level of the counselee was also a significant predictor (β = .59; CI: .32 to .87; *P *= .000). Additionally, counselees who were asked to return for a follow-up consultation recalled less than those who had only one consultation (β = -.46; CI: -.92 to -.01; *P *= .046). And finally, counselees tended to have more recall when they had seen a genetic counselor (nurse) instead of a clinical geneticist (β = .27; CI: .00 to .55; *P *= .047) and less recall when they had seen a counselor who was still in training (β = -.29; CI: -.57 to .00; *P *= .048). This was not related to the total number of information items discussed (geneticists M = 7.01 SD = 2.45; counselors M = 6.93 SD = 2.56).

**Table 6:** Counselees' recall of information items concerning topics discussed in the consultation.

	UC group (*n *= 94)			Intervention group (*n *= 103)				
	**N items discussed**	**Recalled items**	**% items recalled**	**Discussed**	**Recalled items**	**% items recalled**		

	**M (SD)**	**M (SD)**	**M (SD)**	**M (SD)**	**M (SD)**	**M (SD)**	***P* ^a^**	***P* ^b^**

Total	6.79 (2.43)	3.17 (2.07)	45.43% (21.98)	7.12 (2.55)	3.49 (2.28)	49.64% (24.45)	.10	**.02**

Topics (items)	N (%) ce topic discussed	M (SD)		N (%) ce topic discussed	M (SD)		***P* ^a^**	***P* ^b^**

Probability that hereditary breast cancer runs in the family	84 (100)	.93 (.30)		91 (97)	.90 (.45)		.90	.85
Possibilities DNA-test	82 (97)	.78 (.46)		88 (95)	.80 (.45)		.11	.78
Limitations DNA-test	77 (92)	.66 (.58)		82 (89)	.78 (.67)		.50	*.09*
(the risk of hereditary bc can not be ruled out, testing only performed on affected individuals, unclassified variant)								
Possibilities for early detection of breast cancer	77 (93)	1.00 (.85)		88 (95)	.89 (.98)		.51	.76
(mammography, MRI, ultrasound, breast self examination, clinical breast examination of GP/surgeon)								
Possibility of risk reducing breast surgery	25 (30)	.48 (.51)		43 (46)	.68 (.52)		**.04**	.15
Emotional consequences of genetic counselling	47 (57)	.73 (.73)		60 (65)	.80 (.67)		.82	.85
(for the counselee and/or for relatives, for example being reminded of the illness period, feelings of guilt towards relatives, possibilities for support)								
Involving family members in the genetic counselling procedure	68 (82)	1.01 (.50)		82 (88)	.95 (.44)		.75	.58
(Asking for permission to request medical file, asking cooperation for DNA-test, informing about DNA-test)								

^a ^Between group differences for items discussed; ^b^Between group differences for items recalled. bc, breast cancer; ce, counselees; GP, general practitioner; MRI, magnetic resonance imaging; UC, usual care.

In almost all visits, the counselor provided information about the probability that hereditary breast cancer runs in the counselee's family and of the possibilities and limitations of DNA testing (Table 6). The possibility of risk reducing breast surgery was significantly more often discussed in intervention group visits (*X^2 ^*= 4.81; *P *= .03). The probability that hereditary breast cancer runs in the family was recalled best and information about risk reducing breast surgery and the emotional consequences of genetic counseling had the lowest recall scores.

### Knowledge of breast cancer and heredity

Intervention group counselees had relatively more post-visit knowledge of breast cancer and heredity than UC group counselees (β = .30; CI: .03 to .57; *P *= .03; d = .28). Additionally, counselees in whose family there was an indication for DNA testing had more post-visit knowledge (β = .72; CI: .31 to 1.15; *P *= .001). In the intervention group, knowledge especially concerning inheritance and penetrance of *BRCA1/2 *mutations was enhanced (Table 3).

### Needs fulfilment

As shown in Table 4 the intervention group counselees had higher fulfillment scores concerning their cancer genetic information needs (β = .31; CI: .03 to .60; *P *= .03; d = .22). Intervention group counselees especially indicated higher fulfillment of their need for information about the determination and meaning of being a carrier of a mutation in one of the breast cancer genes (β = .29; CI: .01 to .56; *P *= .04) and about hereditary breast cancer than the UC group counselees (β = .42; CI: .12 to.72; *P *= .006). Counselees in both groups reported high fulfillment of generic needs (β = -.18; CI: .36 to .12; *P *= .22).

### Risk perception

Intervention condition was not associated with the alignment of the counselee's perception of her breast cancer risk with the counselor's risk estimation (β = .07; *P *= .79). Table 5 shows the mean difference between counselee and counselor's risk estimation. Neither was there an intervention effect on the perceived relative risk or the verbal indication of the height of the risk of developing breast cancer. Most counselees (101; 67.3%) overestimated their risk of (re-)developing breast cancer post-visit. On average their estimation was 21.62 (SD = 17.42) percentage points higher than that of the counselor. A minority of 40 counselees (26.7%) underestimated their risk with a mean of 10.83 (SD = 8.08) percentage points. The alignment of counselees' risk perception with counselors' estimation did improve for counselees who did not receive an indication for DNA testing, regardless of group allocation. While at baseline 68.8% of counselees overestimated their breast cancer risk based on the risk categories, this was 32.7% post-visit.

Most counselees (75; 48.7%) also overestimated the risk of hereditary cancer running in their family, (average overestimation of 25.68 percentage points (SD = 17.84)) and their risk of being a carrier of a *BRCA1/2 *mutation (92; 61.3%; average overestimation of 23.46 percentage points (SD = 18.66)). Other counselees underestimated these risks (69; 45.4%; mean 16.90 (SD = 13.70) and (52; 34.7%; mean 14.89 (SD = 12.69), respectively). The alignment of these risk perceptions with the counselors' estimations was not significantly associated with the intervention condition (β = .01; *P *= .91 and (β = .07; *P *= .57, respectively; not shown in Table).

### Anxiety

For the whole group of counselees, post-visit anxiety was unrelated to the intervention condition (Table 5). Overall explained variance was 48% and 4% of the variance in the model was due to counselor variation. However, the group of counselees who did not receive an indication for DNA testing (*n *= 49) had significantly lower anxiety scores in the intervention compared to the UC group when controlled for baseline values (β = -.60; CI: -1.12 to -.09; *P *= .02).

### Perceived personal control

Perceived personal control was not significantly related to the intervention condition (Table 5). Levels tended to be higher if there was an indication for DNA testing for the counselee or a family member (β = .34; CI: .01 to .69; *P *= .06).

## Discussion

This study showed that a pre-visit educational website with QPS improves counselees' recall of information discussed in their first visit for breast cancer genetic counseling. As counselees' transfer of information from the visit to relatives has been described as a whisper game where the counselor's information fades out [36], our finding of less noise in counselees' recollection of information is very important. Additionally, counselees considered their need for information better addressed after the visit. Furthermore, we confirmed previous findings that pre-visit education improves breast cancer knowledge [18-20]. These findings are in line with the theoretical notion that provision of pre-visit information combined with increased adjustment of information to the individual increases recall.

In 45-minute first consultations for breast cancer genetic counseling a large amount of information is transferred with the intention that the counselee will understand and remember this information so as to make decisions about DNA testing and to involve relatives [37,38]. This study is the first to assess how much counselees actually remember and found that less than half of the information was recalled. This percentage is similar to levels of recall in oncology outpatient settings [7]. The intervention effect on recall was strongest for those counselees who did not receive an indication for DNA testing and will therefore not have a second visit. Although the effect size was modest, other interventions have failed to produce significant differences [17] or produced small effect sizes [10]. Future endeavors should determine ways to further increase recall.

Effects of the intervention on anxiety were only found for counselees who did not receive an indication for DNA testing. The lack of improvements for those who received an indication for DNA testing is understandable as the indication itself and waiting for the test results can be a source of distress [39]. For counselees who did not receive an indication, their counseling is limited to one visit and they are generally at population risk or slightly increased risk. A decrease in their anxiety is therefore appropriate. Apparently, when counselees had learned about breast cancer and heredity through the website they were better able to process the reassuring information in the visit. The computer-tailored information on the website about indications for hereditary breast cancer and about the need for an indication for DNA testing might have been helpful to prepare the counselee for the population risk estimate. This would result in lower cognitive dissonance during the visit, which contributes to enhanced processing of information [40]. Additionally, they might have better processed the reassuring message because of the slight increase of counselee-specific information in the first visit due to the QPS [25]. QPS studies have found mixed effects on anxiety [10,41]. Possibly, the QPS in the current study showed effects because the questions were sent ahead to the counselor and were endorsed by the counselor.

The pre-visit web-based education had no effect on alignment of counselees' risk perceptions with the counselors' estimation. An explanation for this lack of effect might be the fact that the risk perception, as opposed to factual recall of information, seems to be determined to a large extent by personal experiences of loss [42], identification with affected family members and personality factors [43]. Counselees' perception of their risk of developing breast cancer may therefore be less open to change [44].

Additionally, there were no intervention effects on perceived personal control. Effects of web-based information alone might be limited to cognitive outcomes and might therefore not include perceived personal control [11,45]. In this study, effects on personal control were expected through provision of more counselee-specific information in the visit, but this improvement was small [25]. Most counselees only receive estimations for their personal risk in the final visit when the results of the DNA tests are discussed. Improvements in personal control might thus be more likely after this final visit as only after receiving advice for surveillance or preventive options can counselees take the required actions to control their risk [32]. Additionally, counselees who did not receive an indication for DNA testing for themselves did not gain increased control over decisions. Research on the effects after the final visit is needed.

Analyses were performed with multilevel analysis to take differences in counselor styles into account. This study is the first to show the percentage of variance at the counselor level and this might provide insight into the extent to which differences in individual counseling styles affect genetic counseling outcomes. Although differences between counselors have not been studied before with appropriate methods, several authors have mentioned the need for this [37,44]. For example, geneticists and genetic counselors have received different training and might have different counseling styles resulting in better or worse outcomes. Our study detected a significant difference in the recall of counselees who were counseled by a genetic counselor compared to a clinical geneticist. However, the number of counselors (14) is too small to guarantee reliable effects for variables at the counselor level [46]. The variation in counselors' communication styles and its impact on outcomes should be the focus of future multi-center research allowing for inclusion of more counselors.

The first visit for breast cancer genetic counseling has been described as an educational session in which large amounts of standard information are being transferred and the counselee's understanding is scarcely checked upon [37]. This finding has been reported not only for the Dutch situation [38], but also for the USA [47,48], UK [49] and Australia [47,50,51]. Therefore, we expect that the reported benefits of a pre-visit educational website are generalizable to other countries. However, countries have different health care systems due to which populations of breast cancer genetic counselees and their genetic knowledge might vary slightly [52]. Pre-visit educational websites should therefore be adapted to country-specific settings and populations of counselees.

### Limitations

There are some limitations. First, counselors were not blinded to group allocation as they received counselees' question sheet (QPS) and their responses to these questions were part of the intervention. Second, the response rate is moderate, but relatively high for studies using video recordings of genetic counseling visits [5,38,53]. Importantly, there were no significant differences between responders and decliners and the results of the study are therefore representative for breast cancer genetic counseling counselees. Third, the knowledge scale showed a clear ceiling effect. On at least two of the items hardly any improvements from baseline were possible and this might have hampered the effect size. Fourth, the high percentage of missing values on counselees' risk perception was due to a technical error in the web-based questionnaire and is therefore unlikely to be related to counselee characteristics. Fifth, as we have studied the effects of a combined intervention, we can not distinguish between effects of the two components of this web-based intervention: tailored information and the QPS. Both the fact that counselees learned from reading information on the website and the endorsement of the QPS in the visit might have contributed to the reported effects. Sixth, this study lacked power to untangle gender differences in counselor communication.

## Conclusions

When counselees had prepared with a pre-visit website, they remembered more information from their first consultation for breast cancer genetic counseling and their information needs were better addressed. If adopted in practice, pre-counseling education could lead to more effective first visits for breast cancer genetic counseling due to improved cognitive outcomes. Counselees who need to transfer information to their family might better succeed as a result of increased recall of what was discussed with the counselor.

## Abbreviations

*B*: beta; BC: breast cancer; CI: confidence interval; d: Cohen's effect size; GP: general practitioner; ICC: intra class correlation; M: mean; MRI: magnetic resonance imaging; N: number; P: probability; PPC: perceived personal control; QPS: question prompt sheet; QUOTE: Quality of counselling Through counselees' eyes questionnaire; RCT: randomized controlled trial; SD: standard deviation; STAI: State-Trait Anxiety Inventory; UC: usual care; UMC: University Medical Center.

## Competing interests

The authors declare that they have no competing interests.

## Authors' contributions

AA carried out the acquisition of data, performed the statistical analyses and drafted the manuscript. SvD conceived of the study, participated in its design and coordination and helped to interpret the data and helped to draft the manuscript. JB participated in the design of the study, helped to interpret the data and helped to revise the manuscript. MA participated in the study design and coordination, helped to interpret the data and helped to revise the manuscript. All authors read and approved the final manuscript.
